The article "miR-519d downregulates LEP expression to inhibit preeclampsia development" was retracted in 2022. Reasons: errors in the images; duplicated images; signs of a paper mill.

# miR-519d downregulates LEP expression to inhibit preeclampsia development

**DOI:** 10.1515/med-2021-0244

**Published:** 2021-08-25

**Authors:** Hairui Cai, Dongmei Li, Jun Wu, Chunbo Shi

**Affiliations:** Obstetrics and Gynecology Department, Ningbo Women & Children’s Hospital, No. 339, Liuting Road, Ningbo 315000, Zhejiang Province, People’s Republic of China

**Keywords:** microRNA-519d, leptin, preeclampsia, trophoblast cells

## Abstract

The purpose of the current study was to characterize role of microRNA (miR)-519d in trophoblast cells and preeclampsia (PE) development and its potential underlying mechanism. Regulation of leptin (LEP) by miR-519d was verified using a dual-luciferase reporter gene assay. Loss- and gain-of-function assays were conducted to detect the roles of miR-519d and LEP in proliferation, migratory ability, and invasive capacity of HTR-8/SVneo cells by means of CCK-8 assay, scratch test, and Transwell invasion assay, respectively. The cell apoptosis rate and cycle distribution were analyzed by flow cytometry. LEP expression was elevated, whereas miR-519d level was suppressed in the PE placenta samples compared with those from normal pregnancy. Depletion of LEP promoted proliferation, migratory ability, and invasive capacity and repressed apoptosis. miR-519d could bind 3′ untranslated regions (3′UTRs) of LEP, the extent of which correlated negatively with LEP expression. miR-519d suppressed the expression of LEP in HTR-8/SVneo cells. Moreover, overexpression of miR-519d promoted survival and migratory ability of HTR-8/SVneo cells. Taken together, we find that miR-519d targeted LEP and downregulated its expression, which could likely inhibit the development of PE.

## 1 Introduction

Preeclampsia (PE) is a common complication of pregnancy, which can in severe cases lead to maternal death [1]. The incidence of PE is approximately 3–5%, and clinical data show that PE is likely to manifest in elevated blood pressure starting at 20 weeks of pregnancy [2]. PE is featured by maternal brain injury and placental dysfunction, leading to impaired viability of the fetus [3]. Abnormal invasiveness of trophoblasts is associated with deficient placentation and is held to be a key factor in the pathogeneses of PE [4]. Timely treatment of PE calls for early diagnosis, which might be obtained through innovations in biomarker molecular medicine. It has been reported that the detection of endothelial progenitor cells (EPCs) and natural killer (NK) cells in peripheral blood of women early in their pregnancy can be used as an effective screening method for risk of PE [5]. The significant changes in the serum markers of early PE (early pregnancy) include increased levels of soluble fms-like tyrosine kinase-1 (sFlt-1), soluble Endoglin (sEng), placental protein 13 (PP13), C-reactive protein (CRP), adrenomedullin (ADM), inhibin A (Inh-A), activin-A (Act-A), leptin (LEP), Th1 cytokines, Th17 cytokines, and M1 macrophage-related cytokines, as well as decreased levels of placental growth factor (PIGF), placental protein A (PAPP-A), Th2 cytokines, Tregs cytokines, and M2 macrophages-related cytokines [6]. Despite the broad range of markers, there are few effective or preventative interventions for PE, and the underlying molecular basis of PE still remains largely unknown. It is therefore relevant to conduct an in-depth study of potential therapeutic targets, which may improve the prognosis of PE.

The article "miR-519d downregulates LEP expression to inhibit preeclampsia development" was retracted in 2022. Reasons: errors in the images; duplicated images; signs of a paper mill.

There are report that microRNAs (miRNAs) are important factors with aberrant expression in PE development [7,8]. miRNAs are an extensive family of small noncoding RNAs that affect various biological processes involving cell differentiation and metabolism [9]. The altered expression of certain miRNAs may play essential roles in various placenta-related diseases, including PE and fetal growth restriction [10,11]. For example, the expression of miR-548c-5p in serum exons and placental monocytes of PE patients is significantly downregulated relative to that in healthy controls, which may have a net anti-inflammatory effect in PE [12]. In addition, PE samples show decreased expression of miR-221-3p, which is an miRNA that promotes growth, invasion, and migration of trophoblasts [13]. Furthermore, miR-519d expression in placental trophoblasts participates in the regulation of cellular migration/invasion in PE [14]. However, the downstream mechanisms of miR-519d in PE remain to be explored. As shown by bioinformatics analysis conducted in our study, miR-519d may interact with LEP. Aberrant expression of LEP has also been identified in PE, suggesting that it may play a role in the onset of PE [15]. Moreover, previous work has documented that the LEP gene is hypomethylated in placenta of PE patients [16]. Previous studies have reported that increased LEP levels in the placenta of patients with severe PE may be caused by placental hypoxia. Thus, the maternal plasma level of LEP may bare some relationship with the extent of hypoxic deterioration placenta in PE. Molvarec et al. found a correlation between the serum levels of LEP and the inflammatory marker CRP. They also observed that the increase of sFlt-1 and the decrease of PIGF were unrelated to the serum level of LEP, indicating independence of these mechanisms in the pathogenesis of PE [17]. Early in pregnancy, the free LEP index (fLI, leptin/leptin soluble receptor) was significantly higher in the PE cases than in the control pregnancies [18]. Based on the above research findings, we speculated that miR-519d may be involved in the occurrence of PE by modulating the biological functions of trophoblast cells in association with LEP. Through our investigation of the role of miRNAs in PE, we attempted to establish better the molecular basis for PE and thus to develop potential biomarkers for PE diagnosis and therapy.

The article "miR-519d downregulates LEP expression to inhibit preeclampsia development" was retracted in 2022. Reasons: errors in the images; duplicated images; signs of a paper mill.

## 2 Materials and methods

### 2.1 Bioinformatics analysis

Microarray data (GSE54618) and annotating probe files related to PE were downloaded from the GEO database (https://www.ncbi.nlm.nih.gov/geo/). We identified differentially expression genes by R language based on the |log FC| > 1, *P* < 0.05 threshold, and depicted those genes by heat map.

### 2.2 Study subjects

In this study, 80 pregnant women were recruited from the obstetrics department in Ningbo Women & Children’s Hospital from June 2016 to October 2018 and conducted follow-ups from the prenatal examination to the end of delivery. Subjects were assigned into a PE group (40 cases) and a normal pregnancy group (40 cases) according to their symptoms and signs. Normal pregnancy was defined as having blood pressure or urine protein in the normal range within 35–40 weeks of pregnancy, followed by caesarean delivery of healthy infants. All subjects were mononucleosis-free and (except for the PE symptoms in the PE group) had no other medical and surgical complications before and after pregnancy. The relevant definitions for PE markers follow the eighth edition of Textbook of Obstetrics and Gynecology [19]. Hypertensive disorder complicating pregnancy is a common but severe complication with symptom that includes transient hypertension (systolic blood pressure: SBP ≥140 mm Hg and/or diastolic blood pressure: DBP ≥90 mm Hg), which often disappears within 12 weeks after delivery; urinary protein is negative. This diagnosis can usually be made after delivery. Mild PE is defined as SBP ≥140 mm Hg and/or DBP ≥90 mm Hg with urinary protein ≥0.3 g/24 h or random positive urinary protein (+) after 20 weeks of pregnancy. Severe PE is defined as continuously increased blood pressure and urinary protein, occurrence of maternal organ dysfunction or fetal complications, and occurrence of any of the following adverse conditions: (I) SBP ≥160 mm Hg and/or DBP ≥110 mm Hg; (II) urinary protein ≥5.0 g/24 h or random proteinuria ≥(+++); (III) persistent headache, visual dysfunction, or other neurological symptoms; (IV) persistent epigastric pain, liver subcapsular hematoma, or liver rupture; (V) abnormal liver function, increased level of alanine aminotransferase (ALT), or apartate aminotransferase (AST); (VI) abnormal renal function: oliguria (<400 mL/24 h or <17 mL/h) or serum creatinine >106 µmol/L; (VII) hypoproteinemia with pleural effusion or ascites; (VIII) abnormal blood system: continuous decrease of platelet and less than 100 × 10^6^/L; intravascular hemolysis, anemia, jaundice, or increased level of lactate dehydrogenase (LDH); (IX) heart failure and pulmonary edema; (X) fetal growth restriction or oligohydramnios. Exclusion criteria in the study were pregnant women with primary hypertension, heart diseases, chronic kidney diseases, hepatitis, diabetes, infectious diseases during pregnancy, or other complications during pregnancy. During delivery, we prepared clean gauze and saline for collecting placental specimens. After cesarean section, a 1 cm cubic portion of placental tissue was collected using a sterilized knife under a sterile environment. Samples were taken around the placental fetal surface and at extending about 2 cm from the root of the umbilical cord, avoiding calcified plaques. Samples were collected within 10 min of the delivery of the placenta and were washed twice with saline and wiped with gauze. One half of the samples were stored at −80℃ for later molecular biological testing, and the other samples were fixed in 4% paraformaldehyde solution and paraffin embedded for subsequent immunohistochemical staining analysis. The study was approved by the institutional review board of Ningbo Women & Children’s Hospital, and all subjects signed an informed consent form.

The article "miR-519d downregulates LEP expression to inhibit preeclampsia development" was retracted in 2022. Reasons: errors in the images; duplicated images; signs of a paper mill.

### 2.3 Immunohistochemical stain

Paraffin-embedded sections were dewaxed 3 times with xylene (10 min each time) and hydrated with gradient alcohol. A newly prepared 3% H_2_O_2_ was dropped onto the slices, which were then washed three times with 0.01 M phosphate buffer (PBS). The slices were soaked in 0.01 μM citric acid buffer (pH 6. 0) at 95℃ for 15 min, and then added with an appropriate amount of serum blocking solution, incubated at 37℃ for 60 min, followed by addition of primary antibody LEP (ab3583, 1:200, Abcam, UK) for incubation overnight at 37°C. After washing 3 times with 0.01 M PBS, we added the secondary anti-IgG antibody (ab205718, 1:1,000, Abcam, UK) and incubated the sections at 37℃ for 20 min. Then the sections were treated with DAB chromogenic substrate, counterstained with hematoxylin, differentiated in 1% hydrochloric acid solution for 2 s, treated with 1% aqueous ammonia, and mounted for microscopic examination. Images from each sample were collected in a double-blind design. Quantitation of immunopositive cells was done under high magnification by counting 100 cells in each of ten randomly selected fields per slide. Those cells containing brownish yellow dots were considered positive. Negative expression was designated for <20% positive cells, positive expression for 20% ≤ positive cells < 50%, and strongly positive expression was positive cell count ≥50%.

The article "miR-519d downregulates LEP expression to inhibit preeclampsia development" was retracted in 2022. Reasons: errors in the images; duplicated images; signs of a paper mill.

### 2.4 HTR-8/SVneo cells cultivation and grouping

HTR-8/SVneo cells were purchased from ATCC company (Article number: MZ-2011; Manassas, USA). The cells were placed in RPMI-1640 medium (Thermo Fisher Scientific, Waltham, USA) supplemented with 10% fetal bovine serum (FBS; Thermo Fisher Scientific), 100 U/mL penicillin, 100 mg/mL streptomycin, and a humidified incubator containing 5% carbon dioxide at 37℃. The simulants and inhibitors of miRNA-519d-3p and corresponding negative controls were purchased from Guangzhou Ruibo Biotechnology Co., Ltd. pcDNA3 and recombinant plasmid pc-LEP were designed and synthesized by Shanghai Gene Pharmaceutical Co., Ltd. (Shanghai, China). LEP shRNAs were purchased from Sigma (USA), the sequences are as following:

LEP-shRNA-1: 5′-CCGGATATATACACAGGATCCTATTCTCGAGAATAGGATCCTGTGTATATATTTTTTG-3′;

LEP-shRNA-2: 5′-CCGGCCTTCCAGAAACGTGATCCAACTCGAGTTGGATCACGTTTCTGGAAGGTTTTTG-3′.

The cell density of each group of HTR-8/SVneo cells was adjusted to 1 × 10^5^ cells per well and inoculated in 6-well cell culture plate (2 mL/well). When confluence reached 60–70%, cells were transfected according to the instructions of the Lipofectamine 2000 kit (Invitrogen, Carlsbad, CA) with triplicates for each group. The cells were collected for analysis at 24 h after transfection.

### 2.5 Clone formation test

HTR-8/SVneo cells in each group were digested with trypsin and collected 24 h after transfection. After counting, the cells were evenly diluted, and 1,000 cells were placed in wells of a six-well plate and cultured for 10–12 days at 37°C and 5% CO_2_. Upon formation of cell colonies, samples were fixed with 4% paraformaldehyde, stained with crystal violet solution for 15 min, and then rinsed with ultrapure water. The plates were placed upside down on the operating table to dry, and the number of HTR-8/SVneo cells colonies was counted by naked eye.

### 2.6 Cell counting kit-8 assay

The proliferation ability of cells was determined by Cell Counting Kit-8 (CCK-8) assay. Transfected cells in 100 µL volumes were inoculated into a 96-well plate with a density of 1 × 10^3^ cells per well. 10 μL CCK-8 reagent was added into each well at 0, 24, 48, and 72 h, respectively, and incubated for 2 h. A multifunctional microplate reader was then used to measure the absorbance at 450 nm.

### 2.7 Transwell assay

The invasive capacity of HTR-8/SVneo cells was assessed using Transwell chambers (24-well inserts; 8 µm-pore size; Millipore, Billerica, MA, USA) precoated with matrix gel (200 μg/mL, BD Biosciences, Franklin Lakes, New Jersey, USA). In brief, 24 h after transfection, 10 μg/mL mitomycin C was applied to treat the cells for 2 h. After trypsinization, the cell pellet was collected, resuspended in medium without serum, and seeded in the upper compartment (1 × 10^5^ cells/cavity); the lower compartment contained DMEM-F12 medium with 15% FBS. Transwell chambers were incubated for 48 h, and the contents of the upper compartment gently removed. The invading cells in the lower compartment were fixed in 4% polymethanol, stained with 0.1% crystal violet solution for 15 min, and washed with water three times. Stained cells were counted and imaged in four randomly selected fields per well using an optical microscope.

The article "miR-519d downregulates LEP expression to inhibit preeclampsia development" was retracted in 2022. Reasons: errors in the images; duplicated images; signs of a paper mill.

### 2.8 Flow cytometry

After 48 h of transfection, HTR-8/SVneo cells were harvested and washed twice with prechilled PBS. A portion of the cells was fixed with precooled 70% ethanol, incubated with 500 μL of malonate (PI) for 30 min, and finally analyzed by flow cytometry (FACSArial I; BD Biosciences, San Jose, CA). A single cell suspension was prepared by mixing 100 µL binding buffer with the other cells to attain a final concentration of 10^6^ cells/mL. After adding 5 µL Annexin V 488 (Telo Fisher HealthCo, Inc., Shanghai, China) and 5 µL PI to each group, cells were stored at room temperature for 15 min and then made up to 500 µL with binding buffer. Finally, flow cytometry (FasraciⅠ; BD Biosciences) was used to detect the early apoptosis rate of cells in five replicate samples for each group.

### 2.9 Reverse transcription quantitative polymerase chain reaction (RT-qPCR)

Total RNA was extracted with TRIzol reagent (Invitrogen) and then reverse transcribed to cDNA according to the protocol of the miRcute miRNA First-strand cDNA synthesis kit (Beijing Tiangen Biotechnology, Ltd). cDNA was subjected to real-time PCR using a SYBR premix Ex TaqTM II PCR kit (Takara, Dalian, Liaoning Province, China) with the ABI 7500 real-time PCR instrument. Quantitation of miR-519d was normalized to U6, and LEP was normalized to GAPDH. The primer sequences are listed in Table S1. Results were calculated by 2^−ΔΔCT^ method.

### 2.10 Western blot

The total protein concentration extracted from placental tissues and cells was measured by the BCA method, and the protein concentration of each group was adjusted to the same concentration. The protein samples were separated by SDS-PAGE, electrotransferred onto a PVDF membrane, and probed with primary antibodies: anit-LEP (ab3583, 1:1,000, Abcam, UK) and anti-GAPDH (ab181602, 1:10,000, Abcam, UK) overnight at 37°C. The next day, immunoblots were visualized with goat anti-rabbit secondary antibody (ab205718, 1:1,000, Abcam, UK) and enhanced chemiluminescence detection reagents. The gray values of target protein bands were analyzed by ImageJ (National Institutes of Health, MD).

The article "miR-519d downregulates LEP expression to inhibit preeclampsia development" was retracted in 2022. Reasons: errors in the images; duplicated images; signs of a paper mill.

### 2.11 Dual-luciferase reporter gene assay

The online prediction software DIANA TOOLS (http://diana.imis.athena-innovation.gr/DianaTools/index.php?r=microT_CDS/index) were used to predict the binding site of miR-519d at the mRNA of LEP. The 3′-untranslated region (3′-UTR) sequence of wild-type and site-mutated LEP was constructed into the pMIR-REPORT™ luciferase vector. 1 × 10^5^ HTR-8/SVneo cells were seeded to each well in a 12-well plate. After 48 h of transfection, the cells were removed from the medium and washed 3 times with PBS. The Dual-Luciferase Reporter Assay System (Promega, Cat. No. E10910) was applied to measure luciferase activities according to the procedures of the manufacturer.

### 2.12 Statistical analysis

All statistical analyses were conducted with the software SPSS 22. 0 (IBM Corp., Armonk, NY), and data shown as the mean ± standard deviation. Enumeration data were analyzed using the *X* ^2^ test and expressed as a ratio or percentage. Unpaired *t*-test was used for comparison of two sets of data. Differences among groups were compared with one-way analysis of variance (ANOVA), and data at various time points were analyzed with two-factor ANOVA. The correlation between miR-519d and LEP levels was evaluated with Pearson correlation coefficient. *P* < 0.05 was statistically significant.

## 3 Results

### 3.1 A comparison of clinical data between normal and PE group

As shown in Table 1, there was no significant difference in age, gestational age, and BMI between the normal pregnancy group and PE group (*P* > 0.05). Compared with the normal pregnancy group, blood pressure (systolic and diastolic pressure) and urine protein in PE patients were higher, and the birth weight of infants was significantly lower (*P* < 0.05).

**Table 1:** Clinical data of subjects

Clinical feature	Normal pregnancy group (*n* = 40)	Preeclampsia group (*n* = 40)	*P*‐value
Age (years)	28.00 ± 3.20	29.95 ± 2.67	0.1536
Gestational day at delivery (week)	36.58 ± 2.64	35.68 ± 2.79	0.1421
BMI (kg/m^2^)	30.82 ± 2.95	31.54 ± 2.89	0.2733
Systolic pressure (mm Hg)	121.38 ± 9.57	161.15 ± 12.23	<0.05
Diastolic pressure (mm Hg)	71.15 ± 5.64	104.65 ± 7.96	<0.05
24 h urinary protein (g)	0.11 ± 0.01	5.07 ± 0.39	<0.05
Infant birth weight (g)	3330.50 ± 367.12	2352.58 ± 218.55	<0.05

Note: unpaired *t*-test, compared with normal pregnancy group, and *P* < 0.05 was considered as level of significance.

The article "miR-519d downregulates LEP expression to inhibit preeclampsia development" was retracted in 2022. Reasons: errors in the images; duplicated images; signs of a paper mill.

### 3.2 Elevated LEP expression in PE placenta

Through bioinformatics analysis of the GSE54618 dataset, we found that many genes were significantly upregulated in the PE placenta, but settled our focus on the LEP gene (Figure 1a). The LEP expression profile was confirmed by RT-qPCR, as shown in Figure 1b, confirming that LEP expression was significantly higher in PE compared to normal pregnancy tissue (*P* < 0.05). As shown in Figure 1c, more abundant LEP immunopositive cells were found in the PE group than in the normal pregnancy group. Finally, we confirmed elevated LEP protein levels in PE placenta through Western blot (Figure 1d).

**Figure 1:** LEP is highly expressed in PE placenta. (a) Differential gene expression heat map of the PE dataset GSE54618; the horizontal axis represents sample number, the vertical axis represents differentially expressed genes, the histogram at the upper right depicts the color step, and each rectangle in the figure corresponds to a sample expression value. (b) The levels of LEP in normal pregnancy tissue and PE placenta tissue were tested with RT-qPCR (Normal = 40; PE = 40). (c) Immunohistochemistry was used to detect LEP positive cells (400×) in normal pregnancy tissue and PE placenta tissue (Normal = 40; PE = 40). (d) LEP protein levels were detected by Western blot in normal pregnancy tissue and PE placenta tissue; * indicates compared with normal group, *P* < 0.5 (the result was measurement data, expressed as mean ± standard deviation, and unpaired *t*-test was used for two sets of data statistics result comparison).

### 3.3 Silencing of LEP promotes proliferation, migration, invasion, and survival of HTR/SVneo cells

Impaired migration and invasion ability of trophoblastic cells is considered to be one of the important mechanisms of PE development [13]. In order to detect the effect of differential expression of LEP on the migratory and invasive capacity of HTR-8/SVneo cells, we silenced the LEP gene and tested for changes of cell functions. We first used RT-qPCR and Western blot to detect the silencing efficiency of LEP in HTR-8/SVneo cells. As shown in Figure 2a and b, compared with the si-NC group, the levels of LEP were significantly downregulated (*P*  <  0.5) in the si-LEP-1 and si-LEP-2 groups; therefore, we choose the more efficient si-LEP-2 sequence for subsequent experiments. Moreover, we also overexpressed (oe) LEP using plasmids and confirmed overexpression by RT-qPCR and Western blot (Figure 2c and d). The viability of HTR-8/svneo cells in each group was detected by CCK-8 assay (Figure 2e), cloning ability was measured by clone formation assay (Figure 2f), and cell cycle was determined by flow cytometry (Figure 2g). The cells’ viability and cloning ability in the si-LEP group were significantly increased than the si-NC group, with more cells in S phase, but fewer cells in G0/G1 phase (*P* < 0.5). In contrast, overexpression of LEP in HTR-8/SVneo cells led to lower viability, cloning ability, and proliferation. We used scratch test to detect cell migration ability (Figure 2h) and Transwell test to detect cell invasion ability (Figure 2i). From the above experimental results, we conclude that LEP inhibits proliferation, migration, invasion, and survival of HTR-8/SVneo cells.

The article "miR-519d downregulates LEP expression to inhibit preeclampsia development" was retracted in 2022. Reasons: errors in the images; duplicated images; signs of a paper mill.

**Figure 2:** Downregulation of LEP expression promotes the progress of HTR-8/SVneo cells. (a) RT-qPCR was used to screen the silencing efficiency of LEP in HTR-8/SVneo cells. (b) Western blot was used to screen the silencing efficiency of LEP in HTR-8/SVneo cells. (c) Overexpression of LEP in HTR-8/SVneo cells was detected using RT-qPCR. (d) LEP overexpression in HTR-8/SVneo cells was detected with Western blot. (e) CCK-8 assay was carried out to determine the proliferation ability of HTR-8/SVneo cells when LEP was overexpressed or silenced. (f) Clone formation assay was carried out to determine the cloning ability of HTR-8/SVneo cells when LEP was overexpressed or silenced. (g) When LEP was overexpressed or silenced, the cell cycle distribution of HTR-8/SVneo cells was tested through flow cytometry. (h) Scratch test was used to measure the migration ability of HTR-8/SVneo cells when LEP was overexpressed or silenced. (i) The invasive capacity of the HTR-8/SVneo cells was detected using Transwell test, when LEP was overexpressed or silenced. (j) HTR-8/SVneo cells apoptosis was measured by flowcytometry, when LEP was overexpressed or silenced; * indicates *P* < 0.05 (the measurement data were shown as the mean ± standard deviation, and unpaired *t*-test was used for two sets of data statistics result comparison; single factor analysis of variance was used for multigroup data comparison; data at various time points were analyzed with two-factor analysis of variance, and the tests were repeated in triplicates).

### 3.4 LEP is the downstream target gene of miR-519d

We predicted the upstream miRNA of LEP with miRanda (http://www.microrna.org/microrna/home.do), miRWalk (http://mirwalk.umm.uni-heidelberg.de/), and DIANA TOOLS websites and selected the intersection through the online website (http://bioinformatics.psb.ugent.be/webtools/Venn/). These analyses suggested that miR-330-5p, miR-519d, and miR-326 are potential regulators of LEP expression (Figure 3a). As miR-519d has been reported to be downregulated in PE [20], we chose miR-519d for detailed study and tested its levels in normal pregnancy and PE placenta tissues through RT-qPCR. As shown in Figure 3d, the level of miR-519d was significantly lower in PE than in normal pregnancy tissues (*P* < 0.5). The correlation between miR-519d and LEP expression was analyzed by Pearson correlation analysis, which showed (Figure 3e) that LEP mRNA expression was negatively correlated with miR-519d expression (*r* = −0.602, *P* < 0.001). RT-qPCR and Western blot were utilized to test levels of miR-519d and LEP in HTR-8/SVneo cells when miR-519d was overexpressed or silenced (Figure 3f–h). Compared with NC mimic group, the miR-519d expression in miR-519d mimic group was significantly upregulated (*P* < 0.5) and LEP mRNA and protein expression were significantly downregulated (*P* < 0.5). Compared with NC inhibitor group, LEP mRNA and protein levels were significantly increased (*P <* 0.5). In addition, the binding site of miR-519d and LEP predicted with bioinformatics website is shown (Figure 3b), indicating that miR-519d can bind to the 3′UTR of LEP gene. The dual-luciferase reporter gene assay was applied to demonstrate whether miR-519d directly regulates LEP by binding to this site. As shown in Figure 3c, LEP-WT luciferase activity was significantly restrained by miR-519d mimic (*P* < 0.5), but LEP-MUT luciferase was not affected (*P* > 0.05).

The article "miR-519d downregulates LEP expression to inhibit preeclampsia development" was retracted in 2022. Reasons: errors in the images; duplicated images; signs of a paper mill.

**Figure 3:** LEP is the downstream target gene of miR-519d. (a) Venn Diagram of miRNA binding to LEP gene predicted by Miranda, mirwalk, and Diana tools. (b) The miRanda website was used to predict the miR-519d and LEP target binding site. (c) Dual-luciferase reporter gene assay was used to confirm the miR-519d and LEP binding site. (d) The levels of miR-519d in normal pregnancy tissue and PE placenta tissue were tested using RT-qPCR (Normal = 40; PE = 40). (e) The correlation between miR-519d and LEP expression in normal pregnancy tissue and PE placenta tissue was analyzed by Pearson correlation analysis. (f) miR-519d gene overexpression in HTR-8/SVneo cells was detected by RT-qPCR. (g) When miR-519d was overexpressed or silenced, the level of LEP in HTR-8/SVneo cells was detected with RT-qPCR. (h) When miR-519d was overexpressed or silenced, the expression of LEP protein in HTR-8/SVneo cells was detected by Western blot; * indicates *P* < 0.05 (the measurement data were shown as the mean ± standard deviation, and two independent samples *t*-test were used in comparison; Unpaired *t*-test was used for two sets of data statistics result comparison; Single factor analysis of variance was used for multigroup data comparison; The correlation between miR-519d and LEP was evaluated with Pearson correlation and the tests were conducted in triplicate).

The article "miR-519d downregulates LEP expression to inhibit preeclampsia development" was retracted in 2022. Reasons: errors in the images; duplicated images; signs of a paper mill.

### 3.5 Overexpression of miR-519d reproduces the effects of LEP silencing to HTR-8/SVneo cells

Having shown that LEP inhibits proliferation and invasive ability and is a target of miR-519d, we next addressed whether overexpression of miR-519d could reproduce the LEP silencing effects on HTR-8/SVneo behavior. The CCK-8 assay was applied to analyze the cell proliferation ability and viability of HTR-8/SVneo cells of each group (Figure 4a). The clone formation assay was utilized to measure the cloning formation ability (Figure 4b) and flow cytometry to measure the cell cycle distribution (Figure 4c). The migratory ability, invasive capacity, and apoptosis of HTR-8/SVneo cells were detected with scratch test (Figure 4d), Transwell assay (Figure 4e), and flow cytometry (Figure 4f), respectively. As shown in the Figure, compared with the NC mimic group, the cell viability, cloning formation ability, migration ability, and invasion of the miR-519d mimic group were significantly increased (*P* < 0.5), but the cell apoptosis rate was significantly reduced (*P* < 0.5). At the same time, compared with the NC inhibitor group, the cell viability, cloning formation ability, migration ability, and invasion of the miR-519d inhibitor group were significantly reduced (*P* < 0.5), but the cells’ apoptosis rate was significantly increased (*P* < 0.5). The above results together indicated that overexpression of miR-519d contributes to the proliferation, migratory ability, and invasive capacity of HTR-8/SVneo cells and inhibits apoptosis.

**Figure 4:** miR-519d overexpression promotes the progression of HTR-8/SVneo cells. (a) The proliferation of HTR-8/SVneo cells after silencing miR-519d or overexpressing miR-519d by the CCK-8 method; CCK-8 assay was utilized to test the proliferation ability of HTR-8/SVneo cells when miR-519d was overexpressed or silenced. (b) Clone formation assay was carried out to determine the cloning ability of HTR-8/SVneo cells when miR-519d was overexpressed or silenced. (c) Flow cytometry was applied to measure the cell cycle distribution of HTR-8/SVneo cells when miR-519d was overexpressed or silenced. (d) When miR-519d was overexpressed or silenced, the migratory ability of HTR-8/SVneo cells was measured using scratch test. (e) The invasion of the HTR-8/SVneo cells was detected by the Transwell test, when miR-519d was overexpressed or silenced. (f) HTR-8/SVneo cells apoptosis was measured by flow cytometry, when miR-519d was overexpressed or silenced; * indicates *P* < 0.05 (the measurement data are shown as mean ± standard deviation, and differences among groups were compared with one-way analysis of variance; Data at various time points were analyzed with two-factor analysis of variance, and the tests were repeated in triplicate).

The article "miR-519d downregulates LEP expression to inhibit preeclampsia development" was retracted in 2022. Reasons: errors in the images; duplicated images; signs of a paper mill.

### 3.6 miR-519d’s effects on HTR8/SVneo cells are depended on LEP

To confirm the above scenario, we conducted further experiments using miR-519d mimic and LEP overexpression plasmid to co-transfect HTR8/SVneo cells. First, the expression levels of miR-519d and LEP in the combined experiment were detected using RT-qPCR and Western blot. The results (Figure 5a and b) showed that overexpression of miR-519d significantly downregulated LEP expression (*P* < 0.05), and that LEP mRNA and protein expression were significantly downregulated (*P* < 0.05). The viability of HTR-8/svneo cells in each group was detected by CCK-8 assay (Figure 5c), cloning ability was measured by clone formation assay (Figure 5d), and cell cycle was determined by flow cytometry (Figure 5e). As shown in figure, the cell viability and cloning ability in miR-519d mimic + oe-NC group were significantly increased than NC mimic + oe-NC group, HTR-8/SVneo cells in G0/G1 phase were significantly reduced, and cells in S phase increased significantly (*P <* 0.05). The cell viability and cloning ability in the NC mimic + oe-LEP group were significantly inhibited, with more HTR-8/SVneo cells in G0/G1 phase, and fewer cells in S phase (*P* < 0.05), and it can be seen that miR-519d mimic significantly attenuated the inhibitory effect of LEP overexpression on cell proliferation (*P <* 0.05). The scratch test was used to measure the migration ability of HTR-8/SVneo cells and their invasion was detected by the Transwell test. The results (Figure 5f and g) indicated that the cell migratory ability and invasive capacity were significantly greater in the miR-519d mimic + oe-NC group than in NC mimic + oe-NC group, but were significantly reduced in the NC mimic + oe-LEP group. It can be seen that miR-519d mimic reversed the inhibitory effect of overexpression of LEP on the migratory ability and invasive capacity of HTR-8/SVneo cells (*P* < 0.05). Finally, the cells apoptosis was detected using flow cytometry. As shown in Figure 5h, compared with the NC mimic + oe-NC group, the apoptosis rate of the miR-519d mimic + oe-NC group was significantly reduced, the apoptosis rate increased significantly in the NC mimic + oe-LEP group, and miR-519d mimic significantly restrained the promoting effect of LEP overexpression on the apoptosis rate of HTR-8/SVneo cells (*P* < 0.05). In summary, the overexpression of miR-519d can reverse the effects of overexpression of LEP on the proliferation, migration, invasion, and apoptosis HTR-8/SVneo cells.

**Figure 5:** miR-519d promotes the progress of HTR8/SVneo cells through LEP. (a) After co-transfected with miR-519d mimic and LEP overexpression plasmid, the level of LEP in HTR-8/SVneo cells was detected with RT-qPCR. (b) After co-transfected with miR-519d mimic and LEP overexpression plasmid, the LEP protein level in HTR-8/SVneo cells was detected by Western blot. (c) After co-transfected with miR-519d mimic and LEP overexpression plasmid, the cell viability in HTR-8/SVneo cells was tested through CCK-8. (d) After co-transfected with miR-519d mimic and LEP overexpression plasmid, the cloning ability in HTR-8/SVneo cells was tested using clone formation assay. (e) After co-transfected with miR-519d mimic and LEP overexpression plasmid, the cell cycle in HTR-8/SVneo cells was detected using flow cytometry. (f) Scratch test was used to measure the migration ability of HTR-8/SVneo cells, which were co-transfected by miR-519d mimic and LEP overexpression plasmid. (g) Transwell test was used to measure invasion of HTR-8/SVneo cells, which were co-transfected by miR-519d mimic and LEP overexpression plasmid. (h) After co-transfected with miR-519d mimic and LEP overexpression plasmid, the apoptosis of HTR-8/SVneo cells was measured with flow cytometry; * indicates *P* < 0.05 (the result was measurement data, expressed as mean ± standard deviation, and single factor analysis of variance was used for multigroup data comparison; Data at various time points were analyzed with two-factor analysis of variance, and the tests were repeated in triplicate).

The article "miR-519d downregulates LEP expression to inhibit preeclampsia development" was retracted in 2022. Reasons: errors in the images; duplicated images; signs of a paper mill.

## 4 Discussion

Trophoblast cells are closely associated with placenta formation, which could conceivably promote PE progression through effects on cellular biological function, and indeed, impaired invasion and migration of trophoblast cells are linked to PE development [21]. The HTR8/SVneo trophoblast cells used in the present study are immortalized human extravillous trophoblasts [22]. Furthermore, we collected and analyzed clinical placenta samples. We found that the maternal mean systolic pressure, diastolic pressure, urinary proteins, and the infant birth weight differed significantly in PE patients compared with the normal pregnancy group. Systolic pressure, diastolic pressure, and urinary proteins were significantly higher in PE patients [23]. We next proceeded to conduct a series of experiments to explore the regulatory role of miR-519d in PE. Our results demonstrated that miR-519d plays an inhibiting role in PE development, possibly via effects on the downregulation of LEP.

Initially, we confirmed that LEP was highly expressed in placenta tissues of PE patients. LEP is a hormone secreted by adipocytes, which has shown oncogenic functions in different diseases. For example, LEP aggravates breast cancer by mediating the invasive phenotype of mammary cancer cells [24]. Previous work also attests that, in comparison with pregnant women with normal BMI, PE patients showed higher levels of LEP and proinflammatory cytokines in plasma [25]. Moreover, upregulated LEP secretion can induce perinatal hyperleptinemia, which is one of the characteristics of PE [26,27]. Consistent with our study, it has been reported previously that LEP treatment could regulate placental trophoblast cells by affecting the cellular proliferation, invasion, and nutrient transport [28]. The present new findings illustrated that downregulation of LEP promoted proliferation, invasion, and migration of HTR-8/SVneo cells, but suppressed their cellular apoptosis.

The article "miR-519d downregulates LEP expression to inhibit preeclampsia development" was retracted in 2022. Reasons: errors in the images; duplicated images; signs of a paper mill.

Our mechanistic research further revealed that miR-519d targeted LEP. Burgeoning investigation has confirmed that miRNAs can exert various effects on PE progression [29,30,31]. Similar to our present results, prior work also showed aberrant downregulated expression of miR-519d in PE [14,20]. We now report that forced overexpression of miR-519d could facilitate proliferation, invasion, and migration of trophoblast cells. Consistent with this result, miR-29b also plays a promoting role in the biological functions of trophoblast cells [32], and biological behaviors involving proliferation and migration/invasion are enhanced by overexpression of miR-21 [33]. Although the targeting relation between miR-519d and LEP has rarely been reported, there are some previous works elaborating on the interaction of miRNAs with LEP in PE. For instance, miR-1301 is involved in the regulation of LEP during pregnancy, specifically by negatively regulating the expression of LEP [15]. Other work in the context of gestational disease predicted that LEP could be regulated by has-miR-5699-5p, based on a miRNA-gene network analysis [34].

The results presented above led us to conclude that miR-519d was poorly expressed in placental tissues of patients with PE, whereas LEP was overexpressed due to negative targeting of LEP by miR-519d. Overexpression of miR-519d could downregulate LEP to promote the proliferation and migration/invasion of HTR-8/SVneo cells, hence plausibly hindering the development of PE (Figure 6). This study may provide a theoretical basis for the discovery of miR-based therapeutics against PE. However, we acknowledged that additional mechanisms may participate in the regulation and underlying mechanism of miR-519 in PE, since one specific miRNA potentially may target numerous mRNAs and produce net effects that depend on the presence of both miRNA and its target within a specific cell type. Therefore, a search for additional possible regulatory mechanisms involving miRNAs seems justified. Furthermore, our study entails only investigations *in vitro* and should be supplemented by studies in a rodent PE model.

The article "miR-519d downregulates LEP expression to inhibit preeclampsia development" was retracted in 2022. Reasons: errors in the images; duplicated images; signs of a paper mill.

**Figure 6:** The mechanism diagram of miR-519d regulating PE development. miR-519d was poorly expressed in placental tissues of patients with PE, whereas LEP was overexpressed due to negative targeting of LEP by miR-519d. Overexpressing miR-519d downregulates LEP to promote the proliferation, migration, and invasion of trophoblast cells, thereby inhibiting the development of PE.

## Appendix

**Table S1:** Primer sequences used for RT-qPCR

Gene name	Primer sequence
miR-519d	F: 5′-CAAAGTGCCTCCCTTT-3′
	R: 5′-CAGTGCGTGTCGTGGAGT-3′
U6	F: 5′-CCAUGCUCUUCUACUCCU-3′
	R: 5′-CACUGAUGUCGGUUAGUU-3′
LEP	F: 5'-TGCCTTCCAGAAACGTGATCC-3'
	R: 5'-CTCTGTGGAGTAGCCTGAAGC-3′
GAPDH	F: 5′-CGGAGTCAACGGATTTGGTCGTATTGG-3′
	R: 5′-GCTCCTGGAAGATGGTGATGGGATTTCC-3′
